This article has been retracted.

# Development of Wireless Network Indoor Coverage System Based on Optical Fiber Distribution System

**DOI:** 10.1155/2022/9728536

**Published:** 2022-07-05

**Authors:** Pu Song, Shangkun Xiong, Sen Xu, Jianquan Li

**Affiliations:** ^1^China Telecom Research Institute, Beijing 102218, China; ^2^China Telecom Group Beijing Branch, Beijing 100032, China

## Abstract

With the continuous development of network communication technology, the domestic network has covered the homes of ordinary people, but the indoor coverage system of the network cable network needs to be further improved. The optical fiber distribution system is a signal coverage system integrating GSM, TD-SCDMA, and other standards. It is mainly composed of system access unit, system expansion unit, and system remote unit. Wireless network is an important communication technology, which is easy to use and can be connected wirelessly over long distances. The purpose of this paper is to study an optical fiber distribution system for indoor coverage design of wireless networks, so as to achieve faster and more efficient coverage. In this paper, a wireless network signal processing algorithm is proposed, and a systematic method for designing the wireless network indoor coverage of the optical fiber distribution system is proposed, and the algorithms are compared and tested. The test results in this paper show that the signal strength obtained by the algorithm in this paper is −54.83 dB, while the traditional artificial design algorithm is only −45.97 dB. In addition, the wireless network base point of the algorithm in this paper is also 3 lower than the traditional one. Moreover, the coverage rate achieved by the algorithm in this paper is 3.17% higher than that of the network cable network base point layout given by the genetic algorithm, and the average received signal strength is 3.34 dB higher. In addition, the algorithm in this paper takes 9.1 s, 11.2 s, and 5.3 s for the three scenarios of underground parking lot, large shopping mall, and residential residential area, while the traditional manual design algorithm takes 87.9 s, 108.8 s, and 51.7 s, respectively. The algorithm in this paper is only about 1/10 of the traditional artificial design algorithm. Therefore, it can be concluded that the coverage effect of the wireless network indoor coverage system of the optical fiber distribution system designed in this paper is significantly improved.

## 1. Introduction

Mobile communication services are undergoing significant changes as a result of rapid innovation in communication networks. Ultra-high-speed data and video services can be supported on any network, from the first 2G network to call and SMS services, to later 3G data services, to today's 4G and 5G networks. The demand for high-speed service data is increasing, requiring not only fast access speeds and a large number of users, but also low latency. The coverage requirements for indoor signals are more stringent because the indoor environment frequently has many dead spots. The optical fiber distribution system is an indoor distribution system that uses an optical fiber as the signal's transmission medium, ensuring signal quality, as the three major domestic operators (China Mobile, China Unicom, and China Telecom) will carry out a large number of indoor distribution constructions in urban centers, shopping malls, office buildings, and other places with dense traffic. Moreover, the three major operators build their own indoor optical fiber distribution systems independently, which is likely to cause great waste of resources. In order to solve the problem of waste of resources that still exists, the state has changed the original construction mode of the three major operators by reintegrating the architecture of the indoor distribution system and integrated all the systems of the three major operators into one system.

Controlling indoor wireless coverage is critical for ensuring better reception at the user's location, minimising interference to other wireless systems and lowering the risk of unintended user reception, all of which are critical. Existing solutions are prohibitively either expensive or inconvenient to configure. Furthermore, traditional macrobase station construction can no longer meet indoor coverage scenarios due to the blocking effect of some building materials on radio waves, which increases the difficulty and loss of signal transmission. Furthermore, using a single multiantenna technology to improve indoor coverage is limited and does not fundamentally solve the problem. Currently, using an indoor coverage system to achieve uniform and deep coverage of the indoor environment is a good practise. The following goals should be met in order to build an LTE indoor coverage system: (1) not all indoor scenarios are suitable for the LTE indoor coverage system. As a result, multiple factors such as business needs, performance requirements, investment costs, and retrofit feasibility must be evaluated during construction. (2) While ensuring the quality of the LTE network, the existing coverage system's stability and security cannot be compromised. (3) The indoor and outdoor signals are independent of one another, ensuring that they do not interfere with one another. (4) Other indoor signals, such as 2G and 3G, try to achieve multisystem sharing to avoid signal interference.

At present, 3G and 4G indoor coverage system facilities have been basically perfected, and the coverage, signal quality, and anti-interference ability can also meet people's requirements. However, with the popularization of LTE network, its signal coverage problem has gradually attracted everyone's attention. For some enclosed spaces, entertainment venues with large crowds, and concentrated buildings, the quality, coverage, and capacity of LTE networks are not satisfactory.

Millimeter-wave beam steering is the key technology for 5G wireless communication at present. The 28 GHz and 38 GHz bands are widely considered candidates for 5G. In the context of indoor coverage, fiber-optic wireless systems with multiple base sites that simplify long-range wireless networks are attractive to avoid indoor coverage problems caused by the high penetration loss of mmWave signals. Radio beam steering (and beamforming) is required in order to obtain sufficient wireless network base point gain in the millimeter waveband. Combining fiber-optic wireless systems with remotely controlled photonic millimeter-wave beam steering could lead to significant advances in energy efficiency and cost.

The innovation of this paper is that it summarizes the relevant research conducted by some scholars, so as to understand the development status of the research object in this paper. On this basis, a new algorithm is proposed, and a wireless network indoor coverage system of optical fiber distribution system is designed. In this paper, two algorithms are compared and tested for the system and analyzed in different scenarios.

## 2. Related Work

Regarding the wireless network indoor coverage system, many scholars have carried out related research on it. Among them, Cao et al. explored two indoor fiber-optic wireless network architectures for mmWave beam steering. Cao et al. discussed and studied the key enabling device, the arrayed waveguide grating feedback loop (AWG-loop). Based on AWG-loop, two optical fiber wireless links are further designed to adapt to the two network architectures. Both links with bit rates from 50 Mb/s to 8 Gb/s per spatial channel were experimentally demonstrated at 38 GHz carrier frequency. Cao et al. used an advanced reverse modulation optical transmitter and half-cycle QAM-16 modulation to achieve a record-breaking 16 bits/s/Hz spatial spectral efficiency of its kind [1]. Naqvi et al. introduced a new mmWave access architecture called mmWave over wire (mmWoC). To achieve effective indoor coverage, it features the use of analog modulated relay links to transmit outdoor mmWave signals indoors. Naqvi et al. will discuss the advantages of the proposed mmWoC access architecture and the NC-A2C scheduler, which will be further verified through extensive simulations [2]. Cheng's study investigated the impact of workplace Clean Indoor Air Act (CIAL) coverage on workplace compliance with CIALs, smoking participation of indoor workers, and secondhand smoke (SHS) exposure of nonsmoking indoor workers. Cheng's study estimated several model specifications with and without state or county fixed effects, and the effect of workplace CIAL was consistent across models [3]. Aziz et al. presented empirical IEEE 802.11 indoor coverage and Transmission Control Protocol (TCP) throughput analysis of WLAN access points with corner reflectors. The results demonstrate the potential application of corner reflectors in tailoring indoor coverage and regulating reliable Internet connectivity at access points [4]. The placement of the access point (AP) is an important key to determine the signal propagation range. For optimal signal propagation, network designers need to understand how much coverage an AP can generate. Mukti and Junikhah used coordinate map modeling based on the actual size of the indoor environment to predict the coverage area of the wireless campus network based on AP placement. The results show that the signal generated by the AP will cover the entire area still on the LOS propagation path [5]. PLC (Low Voltage Broadband Power Line Communication) systems transmit their information over power lines over existing infrastructure. However, PLC attenuation and its harsh environment make it difficult to establish reliable communication between the source node and the destination node. The relay-assisted PLC technology can be used to solve this problem to improve the transmission rate and coverage. Zhang et al. conducted research on indoor three-hop relay-assisted PLC system for the first time. Based on a simple PLC attenuation model, the optimal relay node location and transmit power distribution of each node are studied to obtain the theoretical optimal system performance. Zhang et al.'s theoretical work can be used for the design of broadband multihop relay-assisted PLC system and its engineering application [6]. Kafafy et al. investigated the power efficiency of a hybrid RF/VLC indoor system. Kafafy et al. compared the power efficiency of hybrid systems with different layouts of VLC access points. Simulations show that deploying VLC with RF communication can improve the power efficiency of the hybrid system, especially when users receive low RF signals due to walls [7]. Although the research of the above scholars has promoted the development of the wireless network indoor coverage system to a certain extent, most of them are based on theoretical research, either the practical application is relatively small, or the system performance is not perfect and the efficiency is low. Therefore, the research, design, and development of wireless network indoor coverage system based on optical fiber distribution system in this paper are of great significance.

## 3. Indoor Coverage System Based on Optical Fiber Distribution

### 3.1. Optical Fiber Distribution System

Most of the design of the optical fiber distribution system is based on the independent design of each operator, and the standards are not uniform. For today's resource-saving society, it is a design that does not meet the standards. The main research of this paper is to integrate multiple standards into one system. The core of this paper is to develop a new generation of optical fiber distribution system, which is mainly used in the network management design of the system. Because of its unique functionality and applicability, the optical fiber distribution system has been highly recognized by operators in the three years since it entered the market and has been widely used by major operators [8, 9]. These include China Mobile, China Unicom, China Telecom, and China Tower, which have widely adopted this indoor distribution solution.  Figure 1 shows the structure of a traditional fiber distribution system. The structure of the optical fiber distribution system mainly consists of three parts: the access unit, the extension unit, and the remote unit. The access unit mainly couples the downlink radio frequency signals of 2G, 3G, LTE, and other sources, converts them into digital signals and then frames them, and then converts them into optical signals after photoelectric conversion and sends them to the extension unit or remote unit. At the same time, the optical signal in the receiving direction is converted into a digital signal and then deframed and then converted into an uplink radio frequency signal and sent to the source. The extension unit sends the received signal sent by the access unit to multiple remote ends. At the same time, the received signals from more than 45 remote ends are combined and then sent to the access unit. The remote unit converts the received digital signal of the extension unit or access unit into a radio frequency signal in the downlink to realize the wireless coverage of 2G, 3G, and LTE standards. In the uplink, the received radio frequency signal is converted into a digital signal and sent to the expansion unit or access unit.

As a multioperator intensive new optical fiber distribution solution, the multistandard digital optical fiber distribution system is destined to play an important role in the future coconstruction and sharing of rooms with its advantages of high integration and high intensity. In foreign countries, especially in Southeast Asian countries, there are a large number of operators and few frequency band resources. Many of the room subconstructions are led by integrators. After the integrators have done a good job of signal coverage, they are leased to operators, which is similar to the current construction model of China's iron towers. More underdeveloped countries have begun to make similar solutions. From an international perspective, the application range of multistandard digital optical fiber distribution systems will become wider and wider [10, 11].

### 3.2. Wireless Network Indoor Coverage System

In the different stages of mobile business development in the past, operators have had different priorities, whether it was the network that used to be the indoor coverage system, or the channel, or the tariff, the terminal, etc. After passing through a specific period, they have also entered history one after another. The next stage of the development concept is application based [12].

The indoor coverage system construction requirements include requirements to promote the development of the mobile market. Improve the indoor coverage of the mobile communication network by constructing a mobile communication network indoor distribution system. It can help to promote market development and improve the company's brand image, which will help to improve the user's affinity and identity with the network, thereby creating more favourable conditions for the company's market to grow. The brand image is heavily influenced by whether the wireless network can function normally and whether the quality is stable in key locations. The indoor coverage blind area in large- and medium-sized buildings, important underground public places, and high-rise indoor coverage system design buildings is eliminated, and the quality of mobile communication network is improved, thanks to the construction of indoor coverage system. As a result, more people will use the mobile communication network, increasing traffic volume and generating revenue and direct economic benefits. Norms for improving market competitiveness: the company's mobile network's outdoor coverage quality has significantly improved as a result of large-scale network construction in recent years. Improving indoor coverage, improving communication quality, and implementing network optimization have become important measures for some companies to further improve their market competitiveness in indoor areas such as large- and medium-sized buildings, underground public places, hotels, and shopping malls. In sports venues, high-end office buildings, etc., indoor coverage should be used to improve network indicators. Requirements for improving user satisfaction with the growth of users and the expansion of mobile services, users' requirements for network service quality are further improved. How to improve network quality, reduce user complaints, and improve user satisfaction and loyalty are issues that companies must face. It is necessary to optimize and adjust the network in time according to user complaints and network monitoring data. Indoor distribution system is one of the methods to effectively improve user satisfaction [13, 14]. Indoor coverage is a good method, and the composition of the indoor coverage system is shown in Figure 2.

Indoor coverage strategy in the system: one characteristic of the traffic will be the large amount of data traffic. If the main traffic volume in a certain area is the voice service, then the network can completely provide services for users. From this point of view, there is no need to build an indoor distribution system.

The most meaningful classification method [15] for wireless networks is classification by traffic bearer. That is, services are first divided into circuit domain services and packet domain services and then classified according to the bearer rate. The principle of setting up the indoor distribution system is to meet the needs of various businesses from indoors. However, different buildings, scenarios, and different users have different business requirements. It is necessary to choose different equipment types and distribution system types or choose to build in different stages of network development. The following is an analysis of the general business needs of users in different buildings or in different scenarios [16].

It is important to note that the edge bearing rate requirements of different functional areas in the same location are not the same, so a generalised analysis is required. People can use similar business volume to compare the importance of some places. If a building's business volume is high, indicating that users in that building have a high demand for data services, then installing an indoor coverage system in that building is a good idea. On the other hand, if the primary business in a building is voice and the amount of data is minimal, installing an indoor coverage system in that building is pointless. These conditions, of course, are not fixed. Indoor locations with lower data service requirements will gradually increase their demand for data services as network construction progresses. It is necessary to construct an indoor coverage system at this time. The system's main business is data, which is still very different depending on the situation. Users of data services may spend the majority of their time indoors, so this point should be fully considered when designing the indoor coverage system [17, 18]. When designing an outdoor macrocell, services are usually taken into consideration. For the reasons stated above, complete high-speed data coverage for important buildings can be implemented. Traffic statistics can be used to determine the importance of the building designed by the indoor coverage system. The most important buildings should be fully covered, followed by the second most important buildings, which should also be fully covered, and then the rest. Specific user behaviour patterns should be considered when designing the indoor coverage strategy for residential buildings.

At present, it is very common to use the telephone line to surf the Internet at home, and most users have developed the habit of using the telephone line to surf the Internet. It is conceivable that when people need to surf the Internet or download data, the previous habits will continue. Another important factor is price. Relatively speaking, using the telephone line to access the Internet is much cheaper. From this, it can be estimated that, in the initial stage of network construction, the data traffic from residential buildings will not be very large. However, when the network develops to a certain extent, many new value-added services may appear, and the consumption patterns of users will also change to some extent [19].

Because of the relative lag in the development of domestic indoor coverage systems, we are currently in a period of gradual evolution from 2G to 3G, and most buildings did not consider the development needs of 3G when designing indoor coverage systems. As a result, the following issues arise: the standard is not universal, and the repeated construction of coverage systems between different signal standards results in increased noise between systems, frequency band interference, call quality degradation, and a series of disputes with owners. As a result, the focus of indoor coverage system research is on a smooth transformation of the existing wiring system, with the goal of upgrading the 3G system using the simplest methods possible while maintaining the quality of existing network communication. The repeater and WFDS system technologies were developed with the goal of making the system construction method as simple as possible. It reduces the possibility of property disputes while ensuring the quality of system communication and fully considering the needs of subsequent system upgrades to meet the compatibility of multistandard networks [20, 21].

### 3.3. Processing Algorithm of System Wireless Network Signal

For the signal frequency of the system, it can be expressed as

(1) $$\begin{array}{c} f\left(\omega_{1}\right)=A\;\cos\left(\omega_{1}t+\phi_{1}\right). \end{array}$$

Let the local oscillator signal be

(2) $$\begin{array}{c} f\left(\omega_{2}\right)=A\;\cos\left(\omega_{2}t+\phi_{2}\right). \end{array}$$

Then,

(3) $$\begin{array}{c} f\left(\omega_{1}\right)*f\left(\omega_{2}\right)=\frac{1}{2}\left\{\cos\left[\left(\omega_{1}+\omega_{2}\right)t+\left(\phi_{1}+\phi_{2}\right)\right]+\cos\left[\left(\omega_{1}-\omega_{2}\right)t+\left(\phi_{1}-\phi_{2}\right)\right]\right\}. \end{array}$$

Among them, when *ω*_1_=*ω*_2_, this indicates that the signal has completed the baseband conversion.

For the multistage frequency conversion of the system, when the computing resources of the multiplier are insufficient, multiple mixing methods can be used, such as

(4) $$\begin{array}{c} \left(a+bi\right)*\left(c+di\right)=\left(ac-bd\right)+\left(ad\;+bc\right),\\ R=ac-bd,\\ I=bc+ad. \end{array}$$

It can be seen from this that the comb filtering stage after decimation is the main source of delay. Therefore, reducing the decimation multiple of CIC can reduce the delay.

In addition, the frequency word of the carrier output can be expressed as

(5) $$\begin{array}{c} PHI=\text{ROUND}\left(\frac{\theta }{38.4}*2^{32}\right). \end{array}$$

Among them, 32 is the representative bit byte.

For the radio frame length, as shown in Figure 3, it can be expressed as

(6) $$\begin{array}{c} T_{f}=307200T_{s}, \end{array}$$

(7) $$\begin{array}{c} T_{s}=\frac{1}{15000*2048}. \end{array}$$

Among them, *T*_*s*_ represents time.

For the synchronization signal of indoor coverage, it satisfies

(8) $$\begin{array}{c} N_{ID}^{\text{cell}}=3N_{ID}^{1}+N_{ID}^{2}. \end{array}$$

Among them, ID represents the physical layer group of the cell, and *N*_*ID*_^cell^ represents the ID group number.

The position of the synchronization signal in the TDD frame can be shown in Figure 4, and the PSS signal is defined as

(9) $$\begin{array}{c} d_{u}\left(n\right)=\left\{\begin{array}{c} e^{-j\left(\pi n\left(n+1\right)/63\right)},\\ e^{-j\left(\pi un\left(n+1\right)\left(n+2\right)/63\right)}. \end{array}\right. \end{array}$$

Among them, *u* represents the root permutation value.

The sample collection rate in the system satisfies

(10) $$\begin{array}{c} f_{s}=\Delta f*N. \end{array}$$

Among them, *N* represents the sample size, and Δ*f* represents the carrier time slot.

When Δ*f*=7.5 kHz, the regular CP frame is

(11) $$\begin{array}{c} T_{CP}=1024*T_{s}. \end{array}$$

For a sample of *N* points, the zero-padding method is

(12) $$\begin{array}{c} S_{PSS}^{u_{i}}\left(n\right)=\left\{\begin{array}{c} 0,\\ d_{u_{i}}\left(n+30\right),\\ d_{u_{i}}\left(n-\left(N-1-30\right)\right). \end{array}\right. \end{array}$$

Among them, *u* represents *i* root permutations, and *d*_*u*_ represents the PSS signal.

(13) $$\begin{array}{c} n=\left\{N-1,\ldots ,N-1-30\right\}. \end{array}$$

Fractional frequency offset calibration method in the system:

(14) $$\begin{array}{c} {\text{index}}_{i}=m-L_{i}. \end{array}$$

Among them, *m* is the synchronization start position.

The signal is normalized as

(15) $$\begin{array}{c} M_{i}=\frac{R_{i}}{P_{i}}. \end{array}$$

To calibrate the integer octave offset in the system,

(16) $$\begin{array}{c} R\left(k\right)=\sum_{n=0}^{N-1}n^{\prime }\left(n=m\right)e^{\left(-j2\pi nk/N\right)}. \end{array}$$

Among them, *m* is the starting index of the PSS signal (i.e., the primary synchronization signal occupies 6 RBs in the system bandwidth in the frequency domain, i.e., 72sc, indicating the IDPhysical-layerid in a physical cell group). Transform and shift the signal *s* to get the corresponding relationship:

(17) $$\begin{array}{c} S_{PSS}^{\prime }\left(k,s\right)=S_{PSS}\left(\left(k,s\right)\mathrm{mod}62\right). \end{array}$$

By determining the standard sequence, the maximum correlation value index *s* is obtained to estimate the integer frequency offset:

(18) $$\begin{array}{c} F_{0}=s*15\text{ kHz}. \end{array}$$

## 4. Design and Test of Wireless Network Indoor Coverage System

### 4.1. System Design

#### 4.1.1. System Design Goals

A practical wireless network wireless network base point layout design algorithm generally needs to meet the following requirements and enables accurate assessment of coverage performance for a given wireless network base point layout. At the same time, it can give the minimum number of wireless network base points required to cover the designated area and the placement location of these wireless network base points. It is capable of designing large-scale indoor distribution systems. The comparison with the artificial design scheme can be given, so the validity of the design scheme can be verified.

#### 4.1.2. Program Overview

In this solution, the area to be covered is defined as a two-dimensional planar area. The region can be a singly connected or a multiconnected region. To make this problem more tractable, this paper adds two additional constraints: walls and partitions are represented by line segments. For irregularly shaped wall partitions, this paper uses polylines to simulate them. All wireless network base points used in the wireless network base point layout design are omnidirectional wireless network base points, and their transmit power is the same. This is close to the fact that a specific indoor distribution system generally uses the same type of wireless network base point for coverage.

The state of wireless network propagation varies from region to region. The comparison between the prediction results of the underground parking lot and the field test values is shown in Figure 5. The average prediction deviation is 1.42 dB, and the prediction standard deviation is 4.61 dB.

The comparison between the prediction results of large shopping malls and the field test values is shown in Figure 6. The average prediction deviation is 2.24 dB, and the prediction standard deviation is 4.01 dB.

Among them, the comparison results between the prediction results of the residential community and the field test values are shown in Figure 7. The average prediction deviation is 0.21 dB, and the prediction standard deviation is 3.16 dB.

When evaluating coverage for a given area, this paper mainly considers two metrics: coverage and average signal reception strength. In the wireless network design of the wireless network base point layout in this paper, how to use as few wireless network base points as possible to achieve the required coverage in a given area is the most important factor to be considered in this paper. Therefore, this paper regards the coverage rate as the most important indicator of the coverage design of this paper. In addition, maximizing the average signal reception strength in a given area can help improve communication quality. Therefore, this paper regards it as an auxiliary evaluation index. In order to calculate the coverage and average received signal strength generated by a certain wireless network base point layout in a given area, this paper needs to calculate the received signal strength at the positions of all possible receiving points within the given area. In the algorithm, the distribution of receiver points is given by an internal grid of receiver points and by discretizing a given area into a multidimensional grid.

#### 4.1.3. Determination of the Number of Initial Wireless Network Base Points

This paper presents a method to calculate the lower bound value of the minimum number of wireless network base points required to cover a given area. This paper uses a receiver point partition refinement method to calculate. According to the maximum coverage radius of the base point of the wireless network, the receiving points in the center are distributed as evenly as possible to several nonoverlapping cells. The number of cells is the number of required wireless network base points. Here, this paper simplifies the coverage of a wireless network base point to a circle. This is consistent with the assumption earlier in this paper that all wireless network bases are of the same model and transmit power. First, divide the enclosing rectangle into some equal-sized subrectangles. All of the receiving points that fall within the same subrectangle constitute a cell. This gives an initial divided area. Since it may have a relatively complex topology, the above-mentioned initial division needs to be further refined to make the division more uniform. In this paper, a source cell containing very few receiving points is merged into an adjacent target cell. The selection criterion of the target cell is to enable a wireless network base point located at the center of gravity of all reception points in the source cell and the target cell to achieve maximum local coverage in these two cells. After this step, all the receiving points are divided into cells, and each cell needs a wireless network base point to provide services. And the electromagnetic wave penetration loss for the indoor wireless network frequency band is shown in Table 1.

#### 4.1.4. Adjustment of the Number of Adaptive Wireless Network Base Points

In the first iteration of the first phase of this algorithm, this paper calculates a wireless network base point layout optimized by a two-step wireless network base point location optimization algorithm. If the coverage achieved by the optimized location of this wireless network base point is less than the threshold value, this paper also needs to add more wireless network base points in the next iteration. This paper presents an algorithm that adaptively adjusts the number of base points in a wireless network so that the estimate of the pair can be updated at each iteration in-between. The adjustment of the number of wireless network base points can be performed by a fixed step size; that is, one or several wireless network base points are added each time. When using a fixed step size to adjust the number of wireless network base points in each iteration, the actual value can be found by the algorithm as long as it is satisfied. But the step size means more iterations and higher complexity. This paper can reduce the number of iterations when using a larger step size to adjust the number of wireless network base points. But this does not guarantee precise convergence to the actual value. Based on these considerations, this paper adopts the algorithm of adaptive wireless network base point adjustment using variable step size, so that a balance between complexity and accuracy can be achieved. In the multiple iterations of the first stage, the step size for adjusting the number of wireless network base points is adaptively calculated according to the difference between the coverage rate achieved by the wireless network base point layout obtained in the previous iteration and the threshold value. Here, this paper uses two methods to update the estimates of pairs, namely, the method of region resegmentation and the method of quantitative refinement. In each iteration, this paper selects one of these two methods to estimate the number of wireless network base points required for this iteration. The number refinement method uses a step size to adjust the number of wireless network base points each time.

#### 4.1.5. Analysis of Algorithm Complexity

In this paper, the complexity analysis of the wireless network design algorithm for the wireless network base point layout is carried out. This paper presents an algorithm for optimizing the location of the base point of a wireless network using a tree-like simplex algorithm. Considering that most of the computational overhead of the algorithm in this paper is generated by the algorithm, this paper only considers the complexity of the algorithm and the computational cost of the algorithm in the entire design process to simplify the analysis.

### 4.2. Experimental Results

The experiment in this paper mainly includes two parts. In the first part, the design results of the algorithm in this paper are compared with the exhaustive method to verify whether the method in this paper can find a better wireless network base point layout. In the second part, the design results of the algorithm are compared with the artificial design results given by professionals in Zhuhai Mobile Design Institute to demonstrate the practicability of the algorithm in this paper in practical scenarios. Due to the relatively large scene used, this part of the experiment also demonstrates the practicability of the algorithm in this paper in large-scale scenes. In the experiments, this paper will use two criteria to evaluate a given wireless network base point layout. Coverage is the most important factor to be considered in the coverage design of this paper, so this paper takes it as the main evaluation criterion. In addition, the average signal reception strength is also important in coverage evaluation, because it is directly related to the quality of communication in the area to be covered. Therefore, this paper uses it as an auxiliary evaluation criterion. Finally, the number of computations of the objective function is used to measure the complexity of the algorithm, which is in line with previous practice.

In comparison with the traditional manual design, this paper presents the comparison between the coverage design results and the manual design results in the actual scene, as shown in Figure 8. In order to make the comparison meaningful, this paper conducts a drive test in this scenario and corrects the wireless propagation model in the scenario according to the data obtained from the drive test. The corrected results show that the mean value of the error between the predicted value of the model and the measured value is less than 0.47 dB and the standard deviation is less than 5.09 dB, which is in line with the error threshold.

In the experiment, this paper carries out the wireless network coverage design according to the coverage achieved by the artificial design results. In this example, it can be seen from Figure 8 that the wireless network coverage design algorithm in this paper can achieve the required coverage with fewer wireless network base points. Therefore, according to the design results of the algorithm in this paper, the design of the indoor distribution system can greatly reduce the construction cost of the system.

In addition, the performance comparison between the algorithm in this paper and the traditional artificial algorithm wireless coverage layout is shown in Table 2.

It can also be seen from Table 2 that the wireless network coverage rate of the algorithm in this paper is 99.47%, while the traditional artificial design algorithm is only 98.2%. Moreover, the signal strength obtained by the algorithm in this paper is −54.83 dB, while the traditional artificial design algorithm is only −45.97 dB. In addition, the wireless network base point of the algorithm in this paper is also 3 lower than the traditional one.

In the content of the algorithm and the genetic algorithm, the coverage effect of the network cable network base point layout given by the algorithm can be verified according to the comparison of the coverage performance of the network cable network base point layout. The purpose is to compare the coverage ratio and average signal strength achieved by the network cable network base point layout given by the two methods when the same number of network cable network base points is given. Therefore, this paper only optimizes the position of the network cable network base point in the genetic algorithm, and the number of network cable network base points used is consistent with the minimum number of network cable network base points given by the algorithm in this paper. The genetic algorithm library given in this paper can realize the optimization of the base point position of the network cable network based on the genetic algorithm.

This paper conducts comparative tests on several larger scenarios. The experimental results are given in Table 3. The results show that when the number of network cable network base points is the same, the network cable network base point layout obtained by this algorithm is 3.17% higher than the network cable network base point layout given by the genetic algorithm and the average received signal strength is 3.34 dB higher.

In addition, this paper compares the time consumption of the two algorithms for three scenarios of underground parking lots, large shopping malls, and residential buildings, as shown in Figure 9.

As can be seen from Figure 9, the time consumption of the algorithm in this paper for the three scenarios of underground parking lot, large shopping mall, and residential area is 9.1 s, 11.2 s, and 5.3 s respectively, while the traditional manual design algorithm takes 87.9 s, 108.8 s, and 51.7 s, respectively. The algorithm in this paper is only about 1/10 of the traditional artificially designed algorithm, which shows the high efficiency of the algorithm in this paper.

## 5. Conclusions

In the abstract section of this paper, the overall content of the full text is firstly summarized. Secondly, in the introduction, the background of the network era is introduced, the relevant content of the light distribution system is introduced, and the innovation points of this paper are summarized. In the relevant work section, some scholars' researches are cited to understand the current situation of the relevant content of this study. Then, the theoretical research part firstly introduces the optical fiber distribution system, including its characteristics, structure, and related content. Secondly, it introduces the relevant content of indoor coverage system, including its development status, characteristics, and structure. Then, the processing algorithm of the wireless network signal of the system is introduced in detail. Finally, the relevant calculation methods and system design are explained in the experimental part, and the indoor coverage, signal strength, number of base stations, and calculation time of the system are compared and tested. The results show that the system algorithm in this paper is more efficient.

## Figures and Tables

**Figure 1:** Traditional fiber distribution system structure.

**Figure 2:** Composition of indoor coverage system.

**Figure 3:** Frame format.

**Figure 4:** Position of sync signal in TDD frame.

**Figure 5:** Comparison of wireless signal prediction results and field test values for underground parking lots.

**Figure 6:** Comparison of wireless signal prediction results and field test values for underground parking lots.

**Figure 7:** Comparison of wireless signal prediction results and field test values for residential housing.

**Figure 8:** Comparison of wireless coverage layout between the algorithm in this paper and the traditional artificial algorithm.

**Figure 9:** Time-consuming comparison of two algorithm systems in different scenarios.

**Table 1:** Electromagnetic wave penetration loss values in wireless network frequency bands.

Penetration type	Loss (dB)
Grass	5∼8
Ordinary brick-concrete partition wall (<30 cm)	10∼15
Concrete wall	20∼30
Concrete floor	25∼30
Ceiling plumbing	1∼8
Box elevator	30
Human body	3
Wooden furniture, doors	3∼6

**Table 2:** Performance comparison of the wireless coverage layout between the algorithm in this paper and the traditional manual algorithm.

Performance parameters	The algorithm of this paper	Traditional manually designed algorithms
Wireless network coverage	99.47%	98.2%
Average received signal strength	−54.83	−45.97
Antenna required	6	9

**Table 3:** Performance comparison between the algorithm in this paper and the genetic algorithm wireless network coverage layout.

Performance parameters	The algorithm of this paper	Traditional manually designed algorithms
Wireless network coverage	99.47%	96.3%
Average received signal strength	−61.07	−57.73
Antenna required	6	8

## Data Availability

The data used to support the findings of this study are available from the corresponding author upon request.
